The article "Supporting and Studying Organizational Change for Introducing Welfare Technologies as a Sociomaterial Process" was published in 2022. Journal: Front Psychol.

# Supporting and Studying Organizational Change for Introducing Welfare Technologies as a Sociomaterial Process

**DOI:** 10.3389/fpsyg.2022.787223

**Published:** 2022-05-23

**Authors:** Silvia Bruzzone, Lucia Crevani

**Affiliations:** School of Engineering, Business and Society (EST), Mälardalen University, Västerås, Sweden

**Keywords:** welfare technology, sociomateriality, practice, organizational, change

## Abstract

Welfare technologies (WT) for older people is a rapidly expanding sector that offers a way to tackle the challenge of an aging population. Despite their promise in terms of advances in care services and financial savings, their use is still limited. Their design and implementation remain problematic, as they require changes in working practices through coordination among a multiplicity of actors. In order to address these challenges, the need for change is often expressed in terms of a lack of working methods appropriate to their scope. This has led to a proliferation of different toolkits, guidelines, models, etc.; however, these methods often imply a linear understanding of an implementation project and thus fail to take into consideration the emergent and situated character of the processes that lead up to the adoption of welfare. The aim of this article is to propose an alternative means of providing support for the introduction of these technologies by initiating a process for organizational change. The term “change” is understood here as something that is produced by practitioners—in collaboration with researchers—and not brought by researchers to practitioners. To this end, using the tradition of intervention research as inspiration, a learning process at the crossroads of different practices and objects was initiated. The center of attention of this article’ is the sociomaterial process by which different communities of practitioners interact on the co-creation of a checklist. This is a new working method in which the focus is not the artifact in itself but how it emerges through successive interactions and iterations among different objects, practitioners and researchers, resulting in a joint sociomaterial process that reconfigures power relations and the work objective associated with WT. In other words, a new working method artifact is developed in a process in which practitioners, researchers and contextual objects interact and become one with each another.

## Introduction

There has been an increasing focus in recent years on the need to work with change in organizations, in academia as well as among practitioners. The care sector for older people is a particularly interesting context in this respect because it is undergoing profound changes that need to be organized, both within organizations and between organizations and users. Welfare technologies (WT) are increasingly being seen by municipalities as an approach to facing the urgent challenge of an aging population and tackling the severe financial situation in which local authorities are finding themselves. The term “welfare technology” is well-established in the Nordic countries. According to the Nordic Welfare Centre, “Welfare technology is all technology which in one way or another improves the lives of those who need it. The technology is used to maintain or increase security, activity, participation or independence for people with a disability or the elderly.”^1^

Despite its success at a policy level and extensive coverage in the media, the introduction of new WT still presents a major challenge, since it may be that neither professionals or older people use it in the way it was planned by those leading its introduction. As a result, the number of WT that have been effectively implemented remains low (Søndergaard, 2017). Problems arise in the design and implementation of WT (Cozza et al., 2019, 2021), and the lack of systematic approaches and evaluation models may hinder their adoption among operators and management (Baudin et al., 2020). Moreover, although the technologies are publicly funded, we see an unequal distribution among different municipalities (Frennert and Baudin, 2021). The importance of including users (Cozza et al., 2017; Glomsås et al., 2021) is also a central issue. In particular, there is recognition of the need for collaborative approaches in which different kinds of users are made a part of the implementation process from the start, and one central but still problematic aspect is the need to enhance collaboration among different intra- and inter-organizational actors and external actors (such as older people, relatives, etc.) around both the technology to be used and the need to reconfigure organizational practices. In order to tackle this need, institutional actors have proposed a rapidly multiplying variety of implementation tools,^2^ including guidelines, toolkits, models, and platforms.

It has thus been acknowledged that the introduction of WT implies a need to change organizational practices, but there are different ways of working with change. This is often presented as a need to find new working methods and tools, and as we will see later, this was also the case in our study. The methods we have listed above are often linear, however, and organize change as a top-down process. This approach has been criticized by scholars, who have shown that these assumptions of linearity need to be scrutinized, and that change is not easily managed but is a more emergent and organic process than these models imply (Breese, 2011). The aim of this study is to explore an alternative way of providing support for implementing these technologies through collaboration, one that does not take it for granted that a change process is linear, and that involves stakeholders from the outset. In other words, the study explores a process for initiating organizational change in a heterogeneous community of practitioners working with WT. Here, the term “community” is used to refer to “widely dispersed, fluctuating and weakly bounded community forms” (Engeström, 2007, p. 1). It brings together different, yet interdependent, working practices in multiple institutions involved in care work for older people using WT. The intention behind this process is that work should be done *with*, rather than *for*, practitioners.

To this end, a transformative process (Engeström, 1987) was initiated whereby researchers and practitioners were engaged together in producing change in current organizational practices. Beyond a cognitive understanding of working and learning, work is understood in this paper as a sociomaterial (Nicolini et al., 2003; Orlikowski and Scott, 2008; Orlikowski, 2009; Gherardi, 2019) and collective accomplishment that unfolds as an *agencement* (Gherardi, 2019) of human actors, objects and bodies. In this framework, these *agencements* are merely temporary stabilizations of dynamic processes that are constantly under way. The term “change” is understood here as a modification of the *agencement* among the different actors engaged in an experimental project aimed at rethinking collaborative work with WT.

The project takes its inspiration from the method of the Change Laboratory (CL) (Engeström, 1987) which was developed at the University of Helsinki and has the aim of producing the change necessary for a system of activity to evolve. The method is grounded on a conceptualization of work as situated practice, and of learning not as a cognitive achievement but as emerging from the context in which the process unfolds and from local interactions. Hence, knowledge for change is developed within a system of activity, and the role of researchers is to accompany that process. Unlike other methods, solutions are not pre-defined in this approach and the process is not linear, since the method seeks to allow for the complexity and uncertainty of work by encouraging the development of a shared understanding of what the problem is and working together on a possible solution. As we discuss how this method was mobilized in a Swedish municipality, our focus is not on the new working solution in itself but rather on the process whereby human actors and emerging objects interact in an iterative process. This paper is of specific interest to the framework of this special issue as it allows the study of groups in an intervention research context in which practitioners and academics are involved and of the sociomaterial dynamic of co-creation and organizational change.

The article is organized as follows. First the theoretical framework and methodological approach of CL (Engeström, 1987) will be presented, followed by the case study and details of the empirical process. We will then show how we have drawn inspiration from this method in order to give an account of the experimental process applied in a cross-organizational context engaged in adopting WT. The discussion and concluding section will then elaborate further on the overall process of inter-organizational sociomaterial processes in the area of welfare technology, and as a process of co-creation with practitioners more generally.

## Materials and Methods

### Combining the Change Laboratory and a Sociomaterial Understanding of Organizational Practices

The methodological approach adopted in the project takes its inspiration from the experience of the experience of the Change Laboratory (CL), a method developed by Engeström (1987) and colleagues (Engeström and Sannino, 2010; Virkkunen and Newnham, 2013; Engeström et al., 2015; Sannino and Engström, 2017; Nummijoki et al., 2018) at the Center for Research on Activity, Development and Learning (CRADLE) at the University of Helsinki. The method has its origins in cognitive (or social) psychology, in particular in Cultural and Historical Activity Theory (CHAT) (for the origins of the method, see Virkkunen and Newnham, 2013). Since the 1970s, CHAT has made a major contribution to the understanding of human activity as a complex system produced by interactions between an individual subject and his or her community (Engeström, 1987) which is organized by a certain kind of division of labor and by certain rules. Another crucial element of the notion is the idea of mediation, in the sense that an action is always mediated by artifacts that intervene in the performance of the object of the activity and in collaboration with other humans.

At the center of attention for the CL are collaboration, work activities and intervention methods. The method does not focus on an activity in itself but on how it can develop. In this sense, it is a methodology for conducting transformative actions. The first Change Laboratories were implemented in the 1990s. As with other methods of action research, the aim was not to produce observations or knowledge from an external observer’s point of view, but to produce change. As defined by Virkkunen and Newnham (2013), “The CL is a formative intervention method for developing work activities by the practitioners in collaboration with researcher-interventionists” (p. 15). The core idea of the CL is to work on problematic situations in order to produce change in an organizational context. Within this framework, practitioners are considered to be the agents of change, while researchers help accompany the process. Researchers may produce a hypothesis of a solution which is then tried, modified and developed by practitioners according to their experience. The specific aspect of the methodology compared with other methods of action research is that practitioners work on the development of the solution, and not merely on the implementation of a solution that has been developed by researchers (Engeström et al., 2014). The aim of the process is “an expansive reconceptualization of the idea of the activity and reconfiguration of its structure” (Virkkunen and Newnham, 2013, p. 9).

In other words, change is not something that comes out of an external unit—a ready-made, external solution: it happens through a process of reconceptualization of the object of the activity by the participants themselves as part of a learning process. The aim of empowering participants to be the main actors of change (transformational agency) is also integral to the method.

In this framework, the object of the activity is not fixed or given, but depends on the multiple interpretations, understandings and processes of sense-making. The activity is also treated as being mediated by objects that also play a central role in the learning process and the generation of alternatives (Virkkunen and Newnham, 2013). Here, learning is not viewed as a cognitive, individual process: it is inherent in the activity system in which human actors and objects interact.

A central element of the method is the so-called double stimulation (Vygotsky, 1999) which is considered to lie at the heart of agency formation. The first stimulus—which is presented to participants in the form of previously collected mirror data—is a problematic situation, or the main contradiction experienced by actors in their work activity. In the second stimulus, participants are confronted with external artifacts so that they can develop new concepts and alternatives (the zone of proximal development, Engeström, 1987) in order to reconfigure the system of activity (Sannino and Engström, 2017). Contradictions experienced by actors are thus seen as a source for solving problems and learning when interacting on a new object. Learning happens when actors who are experiencing contradictions interact on new alternatives that have the capacity to reconfigure the object of the activity.

In practical terms, the method consists in the organization of a cycle of workshops in which practitioners join with researchers-facilitators to problematize, analyze a working situation and elaborate possible solutions through which the object of the activity is reconceptualized (Virkkunen and Newnham, 2013). The process does not follow a linear logic, in the sense that it is connected to the actors’ iterative process of signification.

In this study, a methodology inspired by CL was mobilized in the area of WT with the aim of demonstrating what it produces in a context that lies at the place where different organizations intersect. In the first phase, the researchers looked for contradictions and tensions that might help the participants frame a problem, and then work on a solution.

It is worth noting the contribution made by Cultural and Historical Activity Theory—from which the CL derives—to the practice turn that since the 1990s has brought about a paradigm shift in the way work, knowledge and learning are understood. In this framework, knowledge is not considered to be a cognitive, individual activity, but one that is intimately inherent in situated interactions within organizational practices. Practices become the loci where learning, organizing and innovation take place (Gherardi, 2019), and there is no separation between working and learning. In this regard, the CL brings an important feature of practice theory: that is, the role played by the materiality in knowing and working. Objects play a crucial role in the execution of tasks and in the material and discursive re-alignment that practice is about. But in this regard, one should note an important difference in the understanding of materiality and scope between CHAT and a stream of theorizing on sociomateriality (Orlikowski and Scott, 2008; Orlikowski, 2009) that foregrounds a relational understanding of reality that is crucial to practice theory (Gherardi, 2019). As Fenwick (2010) points out “The Marxist notion of systemic “contradictions” is central to CHAT, and individual perspectives and interests are constantly at play in negotiating these contradictions. In these features, CHAT retains a more humanist orientation [….]. This human-centric analysis is also evident in the clear delineation of non-human “artifacts” as bounded, distinct from humans, and while embedding cultural histories, are relegated to the role of mediating human activity. CHAT also foregrounds a socio-political analysis of human activity, including constructs such as “division of labor” and “community” (and even social class, prominent in many CHAT analyses), which is anterior to the emergence of elements that may or may not comprise a “system” (Fenwick, 2010, p. 10).

On the other hand, the concept of sociomateriality foregrounds a relational understanding of reality that brings the inseparability of social and material dimensions of practice to the fore. “While an ontology of separateness has long influenced the social sciences—a legacy of Cartesian dualism—its primacy has been challenged in recent decades, particularly through developments in science and technology studies (Barad, 2003). Scholars here have been working within a relational ontology, which rejects the notion that the world is composed of individuals and objects with separately attributable properties that “exist in and of themselves” (Law, 2004, p. 42). This ontology privileges neither humans nor technologies (Pickering, 1995; Knorr Cetina, 1997; Schatzki, 2002; Barad, 2003; Latour, 2005), nor does it treat them as separate and distinct realities” (Orlikowski, 2009, p. 13). In this regard, terms such as “entanglement,” “assemblage” or “*agencement*” (Gherardi, 2019) become relevant to refer to the situated and temporary local encounters of social and of the material.

This means that by leaning on these later developments of practice theories, we build on the CL as a way of working with change, but without distinguishing between the social and the material, or between the subjects and objects of an activity. Rather, we understand subjects and objects as produced through the ongoing assemblage of humans, non-humans, places, routines, etc.

In the following paragraphs we will show how a process of transformational change was initiated at the boundary of different communities of practitioners involved in a process.

### The Case Study

The research took place in a municipality in Sweden that is considered to be fairly advanced in the area of WT, thanks in part to the close connection between the local university and the municipality. This collaboration has resulted in powerful synergies between research and teaching in the area of healthcare and care, on the one hand, and practice and public policies on the other. In Sweden, social services are a right that all citizens possess, and they are delivered by the municipality. In particular, the study focused on the introduction of a camera for remote monitoring at night (often called “the night camera”) as an example of welfare technology. This is one of main technologies municipalities are working with, since there are possible benefits for both municipalities and users if physical visits at night are replaced by digital ones. Digital visits take place in the form of a camera, which is generally placed in the bedroom and is activated a few times every night at specific points in time agreed with the user. Social services personnel can thus monitor the situation from screens in their offices. About 70 night cameras have been activated in the municipality up to today. This has allowed a partial change in the way care services are delivered from night visits to night monitoring (although most visits are still physical or partially physical).

The research process and experimentation presented here has been conducted within the framework of the IVRIS project—which is funded by the national research agency Vinnova—which aims to introduce WT through collaborative practices. The project brought together university researchers and personnel from the municipality—from different units of the care department, including a manager of case officers, homecare personnel (manager and worker), a digitalization manager and a developer—the regional office in charge of disseminating knowledge in the healthcare and care sector (which we will refer to from now on as DISK) and the regional assistive technology center (henceforth RAT), with both a technician and a developer. During the process, two older people who were members of an association for older people were also invited to take part in the workshops so that their perspectives could be included. The municipality has shown a particular interest in this project, and a mid-term report has been presented to the senior management, which is seeking to adopt new ways of working with WT and improving internal coordination among different administrative departments in this area. RAT works mainly with hospitals and people who have just left hospital and need assistive technologies in order to be independent at home, and with other people who need different kinds of assistive technologies. RAT employees thus have an extensive and profound knowledge of technical devices and new technologies, as they are actively looking for new products and understand the technical features of the devices. At the moment, however, there are only limited connections between those municipalities that are responsible for providing welfare services that are at times supported by WT to older people and the RAT. This often results in municipalities adopting solutions with an inadequate insight into the devices’ adaptability for broader local infrastructural systems and professional practices. DISK is at last establishing its role as the main knowledge provider, and is trying to impact municipalities’ choices in terms of WT. In this regard, this research project has been one of the first occasions (if not the first) for bringing all these relevant actors together.

In other words, the project brought together a community made up of different practitioners—both inside and outside the municipality—and older people engaged in WT to initiate a transformative process of organizational change.

In order to be taken into consideration, all these participants were formally partners (except for older people’s association) in the project: that is, they received funding and committed to the project through the research contract required by the funder.

### Empirical Process

Inspired by the CL method described above, “mirror data” were first gathered, mainly through interviews (see the details in the next session).

A cycle of workshops was then organized that brought together most of the people who had previously been interviewed and other representatives of the above mentioned organizations. In these workshops, the participants were invited to interact and exchange their reactions to and reflections on a set of materials (in particular, quotes on practices collected by the researchers during our interviews), in order to analyze actual work practices (not only problems, bottlenecks and contradictions but also strengths) and develop new ideas and tools for changing practices. The work then turned to the development of a checklist. The way the workshops were organized changed as the COVID-19 pandemic affected the opportunities for meeting in person. Three in-person interactive workshops were held, and were attended by an average of 7 to 10 people. Then, owing to the pandemic, two remote workshops were organized with selected informants to tackle the digital format. A third remote workshop was organized with all original participants as a last opportunity to present and discuss the final version of the checklist. The participants in the workshops were a heterogenous group, ranging from senior and middle managers (in the municipality), project managers (RAT and DISK) and personnel at an operational level for the remote monitoring of older people and home care (RAT and municipality). Last but not least, two older persons from an association for older people were involved.

As mentioned above, two sets of data were collected: mirror data from interviews (which ranged from 90 to 120 min) and data from recordings made during the workshops. Both the interviews and recordings were transcribed verbatim and analyzed. The interviews were semi-structured with the objective of identifying bottlenecks experienced by participants in their work with WT. Interviews has been analyzed according to a grounded theory perspective (Charmaz, 2001). In terms of the recordings of the workshops, our analysis focused more specifically on identifying expressions of “transformative agential change” (Haapasaari et al., 2016) specifically connected to the use of WT as it emerged in the process and in interactions with the material support that was given to the participants, in particular extracts from the mirror data, the checklist proposed by the researchers and the final checklist proposed by the participants themselves.

It is worth mentioning that, as developed by CRADLE, the CL is based on ethnographic work and intensive sessions that also require a high level of engagement and time from practitioners. Beyond the fact that it lacked the resources to conduct such a comprehensive study, the project was also particularly affected by a high turnover of the practitioners involved in it (who changed their jobs or areas of responsibility), and above all by the pandemic. This meant that the participants in the process were not always the same, which required a great deal of work by the researchers so that they would be able to provide precise, updated and detailed accounts of the entire process and each workshop to this mobile community of participants. In addition, the time limits imposed by the project meant that it was not viable to follow the implementation of the co-created solution, so it was impossible to give an account of the complete process of organizational change. Within these specific premises and limitations, our work and intervention were inspired by the methodological experience of the CL, which was adapted without aiming to reproduce the specific method in full. What is presented here is thus an example of a sociomaterial process inspired by the CL method, one that is feasible for smaller projects in which the material that can be produced is limited and the opportunity to meet participants is constrained by their work situations, something that is common to many projects and organizations.

What we will see is how the process does not follow a linear dynamic, but has a more iterative movement that is built up in the process through sociomaterial interactions. The configuration of the actors—both human and material—changes during the process as well as their power relations.

## Results

### Collection of Mirror Data

The first step was to collect mirror data to be used in the first workshop to make the participants react and potentially be critical. In particular, preliminary interviews were conducted with the different individuals involved to varying degrees in the process of adopting the so-called night camera in this Swedish municipality. More specifically, interviews were conducted with the municipal managers for quality in the care division (*Vård- och Omsorgsförvaltningen*); the digital strategist from the same division who was responsible for developing new digital solutions for care work; the project manager of the communication, IT and digitalization unit (*Kommunication, IT och Digitalisering Enhet*); and in some case officials (*Biståndshandläggare*) who assess the needs of older people and decide upon each case. Finally, an interview was carried out with the head of the night patrol unit (*Nattpatrullen*), who monitors the older people at a distance and visits them during the night if needed.^3^

Along with these interviews, the researchers were able to build on their observations of meetings of the project group that worked on implementing the night cameras. The researchers also interviewed key informants at DISK and RAT who were indirectly involved in the implementation of the “camera strategy.” It was decided to involve DISK in the design of the process and as the facilitator of the workshops from the very beginning because it already had experience with the subject in the region and with project testing in the WT field (albeit for people suffering from dependencies, for example, rather than older people). The two participants from DISK supported the researchers with making sense of and selecting the material. They also took the role of coordinating some of the workshop discussions. It was also decided from the outset that they would take care of the final results of the process through their website.

The material that was collected and selected involved very different aspects of the practice as a whole. It was organized into a narrative detailing the story of the introduction of the night camera and into different topics. Six challenges were selected from interviewees’ quotes as being specifically meaningful:

1. “There is too much focus on devices”
2. “It does not work to just copy solutions”
3. “Which competences and roles should be included and how? when do we start working with the introduction of WT”?
4. “How can we take advantage of the existing initiatives and competences in the region?”
5. “We do not follow up”
6. “Who should be responsible for the technical objects?”

### First Stimulus—Materializing, Articulating, and Re-materializing

During the first workshop, the participants were introduced to the methodology, and in particular were invited to react to each of the “challenges” selected in the previous phase. The aim of presenting these data was to encourage reactions to a possible definition of the problem or contradictions. Each challenge was presented with longer quotes and projected as a PowerPoint slide on a large screen and discussed individually.

Reactions to each of the challenges were collected on a whiteboard in the form of notes. This material generated intense discussion and the need and motivation to go for welfare technology was not in general questioned by any of the participants during this phase. The contradictions focused on two main problems related to the need for changing organizational practices:

#### Too Much Focus on Devices and an Urgent Need to Better Identify Needs

The focus on devices does not make it possible to think about WT in terms of something that should fulfill someone’s needs. The difficulty experienced by municipal services with working with people’s needs instead of devices and procedures was clearly reported:

“*We often set the structure first, but do not focus much on the person. Where are our users in all of this, where are they? Where are other categories in all of this? Social benefits and things like that, in this? These will often come at a later stage (…). We say: “Now that we have this gadget and this working method, what do you think about it?”. It should be before and say: “How can we solve this [problem] with the resources we have got?.” That is, it is about where to start, where we should start. So, we need to ask them [older people]: “What do you need in order to be more independent?” and then find the right working method and gadget. We are not doing that, but rather saying [to the older person]: “Now we have found something to replace it. Does this make you more independent?*”” (Lisa, head of case office).

#### The Need for New Working Methods in Order to Initiate and Implement Welfare Technologies

What emerged was the problematic nature of the current approaches to WT and the need for new working methods.

“*I’m thinking that when we talk about implementing something, it sounds like it’s all about just starting to use something. But it’s a new way of working and that’s the key issue. It’s not the camera that is important. You need a new way of working; you need a new*… *everyone needs to work differently”* (Julia, case officer).

The question of new ways of working (*artbetssätt*) took different forms and significance depending on the different practitioners. New approaches were also called for in order to pool existing skills at a regional level. The municipality was accused of not taking advantage of existing competences outside its own organization. This was also related to the heterogeneity of the solutions, and a lack of compatibility between some of the devices.

“*We have a technician who works with the door telephone [porttelefoner], but all the municipalities in [name of the Region] have different electronic locks on the doors of their homecares, so it doesn’t work*” (Malin, RAT).

But pooling competences also means integrating users and other internal actors into the process of introducing new technologies. Internal and external actors with relevant skills were not always involved when a new project starts:

“*We forget to train the user and this is why it takes so much time to make him or her use it [the technology]* (Gustav, night patrol).”

It was acknowledged that the organization works in small units, which hinders the initiation of projects that require collaboration from different departments.

Some possible methods or tools to solve these issues and promote change were raised during this phase, and the idea of a checklist was brought up.^4^ This solution was acknowledged and supported by one of the representatives from the association for older people who had worked in an industrial sector where checklists were used extensively.

“*I think the organization is busy delivering a service and what they should do. Then you must have a checklist or some structure or a coach who passes by and recommends how the work should go. Just as we turn to procurement, which knows exactly what to do with procurement, so we have people who work with information security who know “This is what we must do.” We have lots of expertise, but we should use it in the right order. A kind of support that you pick up at*…” (Sara, IT unit).

*“A development plan, an implementation plan. This is how the industry has gone when you think of isonite houses and quality support. Then you have developed a checklist with a number of steps that you must go through, answer, before you can continue to spend money on it. To facilitate decisions and make sure you haven’t missed anything (.) it goes back to the beginning, “Then we have to bring this in at the beginning.” So you always have a process of improvement. I don’t know how it works in the municipality, but I can imagine that it can be very difficult to have an improvement process with things like this there. There are so many people involved. But that’s what you have to work with*” (Sven, association for older people).

Other potential tools were also mentioned in this phase: guidelines, implementation plans and standard guidelines developed by public authorities.

*“You also have autonomous municipalities in Finland, but there is a State that says “You must follow this standard, then you can buy whatever products you want.” I think the remedies are needed in Sweden as well, and it will probably come, but it will take time”* (Peter, DISK).

The lack of a method did not emerge as something completely new: a participant from the IT Department mentioned that the municipality was already working on a project/change management tool inspired by the Benefits Realization Management (BRM) approach. She is also the project leader for developing this tool.

*“The Swedish Financial Management Authority has something called DIGG [Agency for Digital Government], the people who are responsible for digitalization at government level. They have developed a method called the benefit realization template.* (…) *You specify the need when you find it, and you look and estimate what qualitative and economic benefits you have. You also look at when and in what way to follow up the effects. So it is a method, an aid in the introduction of something. I think that’s what we need, we need something to hold on to and we all need to work the same way.”* (Sara, IT unit and project manager of BRM at the municipality).

In this phase, a multiplicity of critical aspects and practices emerged associated with the current design and implementation of WT. The discussion that began from the mirror data was a way of reinforcing and expanding what had been done by the researchers with the mirror data. From the beginning, it seemed that the night camera was not at the heart of the discussion, which rather focused on the need of new working practices (*arbetssätt*) and tools. The camera was cited to give an example of some of the methodological problems (fragmentation among departments), bottlenecks in the procedures (the constraints set by the bid) or the technology itself (the rapid aging of technology, which increasingly leads to leasing solutions).

In this phase, the researchers brought certain issues to the fore by selecting them and producing slides with quotes that justified why they were important. At the same time, the researchers used these slides to approach the style of language used in organizations. The representatives of the different roles and organizations recognized themselves in the quotes and articulated and expanded on the issues. They seldom disagreed; rather, they added to the complexity by building on their own experiences and recounting the issues from specific points of view.

The older people mobilized not only the knowledge they had developed as clients of the municipality, but also knowledge and experiences from their professional lives, for example how things are done in industry. The knowledge they articulated in this way was based on experience, and referred to concrete situations; it was not just about abstract principles, but addressed the situatedness and sociomaterial nature of care practices (Cozza et al., 2019). To try to facilitate an open discussion, the researchers and DISK asked questions and follow-ups, while at the same time retaining the power to materialize what was being said by writing notes on a whiteboard.

### Workshop 2: Further Explorations of the Possibilities for Organizational Change

In workshop 2, the participants were asked to work in pairs (from different organizations or departments) and to discuss specific bottlenecks and challenges from their specific professional perspectives when designing or implementing WT. For the most part, they worked on matters they believed needed to be addressed. Figure 1 shows the material that was produced. They foregrounded the importance of collecting and following up initiatives in banks of ideas. The first group worked around a system of ideas on how to collect, take care of and build up around ideas or initiatives in the area of WT; who can propose ideas or initiatives; and how to collect and store ideas from a multiplicity of sources (from a management group, from operational staff, from older people, from their families or from another municipality).

**FIGURE 1:** Contribution of the different groups to the discussion on bottlenecks and challenges from their specific professional perspective.

The second group worked on certain principles that were lacking or that were important when starting a project or idea, such as perseverance, the right driving forces or brave, systematic or usable ideas. The third group focused on collaborations among different actors (users, personnel and the municipality) as well as on the benefits these actors would derive from the changes to be made. A fourth group discussed who the person leading the process should be, and concluded that the manager was not always the right person: “*Where to go with the idea so that is not “killed” by the wrong person? The manager may not be the best person.*” It was also debated how to better cooperate internally and with external organizations.

In the second part of the workshop, the focus moved once again to possible solutions. As we have already mentioned, the need for a method—and in particular the idea of checklist—had emerged in the first workshop, and so in the second workshop, the researchers prepared different types of checklists for the participants as examples of possible tools (Figure 2). Checklists have already been used in highly complex organizational contexts such as the medical sector (Gawande, 2011) or in the reorganization of social services (see for example the experience of Community Labs in the Region Emilia Romagna: https://www.secondowelfare.it/governi-locali/regioni/welfare-di-comunita-le-innovazioni-che-vengono-dallemilia-romagna/) based on a simple “do not forget” principle. In other words, the aim of checklists is to tackle the complexity of organizational work and keep together all the threads of a practice that may exceed the one single organization, as in the case of the design and supply of welfare services. The researchers showed different types of checklists and asked the participants to develop their own according to what they saw as being important to “remember.” They also asked them to add what had emerged in the first part of the workshop to their checklist (Figure 3). The participants were asked to work in three groups to prepare their own proposals (Figure 3).

**FIGURE 2:** Examples of checklists shown at the workshop.

**FIGURE 3:** Participants’ first draft of checklists.

In the first case, the idea of developing an application to collect and follow new ideas was raised. In the second case, there was an attempt to identify specific phases: documents on decisions, a pilot study, a prototype, a field test and a decision on broad implementation. In the third case, there was an attempt to keep the idea of a checklist with different tasks, phases and comments, and a space to check what had been done.

The initial focus of this second workshop was to expand the participants’ experience of the process of adopting WT (using the example of the night camera), and in particular of disturbances or problems they had encountered in their own work practice. It turned out, however, that things did not work that way. Participants’ focus in this phase was on what should be done, or what general aspects should be taken into consideration to improve the situation, instead of digging into their own professional experience. The tendency was to produce a narrative of the problem and bottlenecks from a general perspective and not from one that was specifically problematic from their own standpoint. It is from this view—on a general level—that they began to identify a number of desirable elements that should become part of (a) possible solution(s).

In this regard, there seemed to be a need to nurture new ideas so that they were not overlooked or killed, given that new ideas can come from different people inside or outside of the organization, and that there is no systematic way of supporting and working with new ideas. It also became clear that the participants envisioned a way of working that made good use of all the knowledge and experience that was distributed across a variety of actors who may not have been in contact with each other at that time.

### Second Stimulus: The Researchers’ Checklist for Guiding Organizational Change

After the attempt to expand the participants’ experiences and understanding of the situation, the aim of the third workshop was to move forward and begin to explore a possible solution and therefore make advances in the proposal of a second stimulus.

First of all, as described above, a project/change management tool was mentioned in the first workshop by one of the participants, who is also in charge of developing it in the organization (we have called her Sara for the purpose of this article). The researchers therefore decided to explore this tool in greater depth in order to discuss how it might be connected to the ongoing process of intervention research. Benefit realization management (BRM) was being tried out at the IT and Digitalization Unit as a planning tool for new initiatives. A search in the literature revealed that it is extensively used by organizations even though it is viewed as being somewhat rationalistic as a tool, and not a true representation of the complexity of organizational life (Breese, 2011). In the third workshop, therefore, BRM was presented by Sara (the IT Unit and BRM project manager). Sara has a background as a project manager for IT projects and has developed her own version of BRM combined with other planning models. Her tool is therefore made up of two main phases, “understand” followed by “create,” inspired by the Double Diamond Model.^5,^^6^ The former- understand- is understood as an investigation phase to collect information, documents, competences and eventual approval of an initiative, while the latter- create- is conceived as the production (of a solution but also of needed contracts, bids, etc.) and implementation phase (including trainings and change management).

The reactions to BRM were very positive, as it was perceived as an attempt to systematize the process and to deal with different initiatives that might be developed over the course of time.

Joan (RAT): *You talked about pausing the other items. They’re not thrown away right away? And that is where they might sit for a while until there are more pieces that might fit together?*
Sara (IT unit and BRM project manager): *Yes.*
Joan: *That’s smart!*
Sara: *And I’m also thinking that if we do that at the healthcare administration, what if the municipality, with their overall view, could have the signals that “We are thinking about this.” I’m thinking, we’re talking about the healthcare administration, but if you look at projects for Smart [name of municipality] or Smart stad there is a fair chance we will develop neighbouring technologies.*

It is worth noting that when the researchers decided to expand the tool and have BRM presented at one of the workshops, they did not know what role it would assume in the ongoing intervention-research process. But as we will show, from that time on, BRM became a part of the discussions and was connected to the checklist, which was the researchers’ second stimulus, so in a way, the second stimulus turned out to be two—the checklist and BRM—instead of one.

Based on what had been developed in the previous workshop, in the second part the researchers proposed a draft checklist developed around the specific case of the camera (see Table 1). This represented the second stimulus, which was meant to make participants analyze the problem and reflect on a possible solution.

**TABLE 1:** First draft of a checklist by the researchers.

Short description of the new solution	Night monitoring service for elderly people through night camera			
Elements of the arbetssätt	Questions	Yes/No	Possible actions	Notes (actions done; specific bottlenecks, etc.)
**Organization as a whole**	Are the benefits for the organization been clearly set?		If yes, specify.	
	Does this contribute to organization mission (uppdrag)?		If yes, specify how? If not, check with Biståndshandläggare, hemtjänst, nattpatrullen	
	Do the different parts of the organization have the resources/competences to put into the process?		If, yes specify. If not known, check with Biståndshandläggare, hemtjänst, nattpatrullen	
	And does this need further specification of the organization or professional groups mission?		If yes, please specify…	
	Is there another way of fulfilling the mission in regards to these needs?			
	Are there any specific competences that need to be developed		If yes, please specify…	
**Organization/Internal users**	Are all parts of/affected by/can affect of the arbetssätt been involved?			
	Has the Bistånd been involved?			
	Has the IT department been involved?			
	has the development department been involved?			
	Has the home care been involved?			
	Has the communication department been involved			
	Are there others that need to use the technology used in the arbetssätt?			
**External-users (for instance older people, relatives)**	Have potential users been involved?		Older people already users, relatives of users, potential users,	
	Have elderly’s relatives been involved?			
	Have elderly people associations been involved			
	Has homecare personnel been involved?			
**Technology**	Is it already used internally otherwise, and could it be used for this too?		Check IT department, etc.	
	Is it already used externally and how?		Check other municipalities, Hjälpmedelcentralen DISK, 4M samarbete	
	Is the technology tested or validated? (for example pilot tested in other municipalities, in research studies or in evaluations)			
	Do other solutions exist on the market?		Check DISK, RAT, Older people associations	
	Is it user-friendly?		Test Collect others’ tests Check Older people associations, current users, FoU	
	Is it easy to maintain?		Check DISK, RAT	
	Do does it need to interact with other systems/apps?			
	How secure does this needs to be?			
	has an option been provided in case of fail?			
**Legal infrastructure**	Are there legal restrictions or requirements?		Check with the Bid service	
**Budget**	Is it possible to insert this action into the current budget ?		If yes, specify which line of budget If no, please specify	
**Other departments**	Does the new solution affect other departments?			
**Other organizations**	Does the new solution affect other organizations?		If yes, which ones	
**Does this generate new ideas regarding other arbetssätt?**				

The researchers’ checklist first distinguished areas inside and outside the organization, and then a multiplicity of questions that were not to be forgotten and were to be answered by a “yes” or “no,” possible actions to be taken and some space for notes. They attempted to condense all the possible questions and issues that had emerged in the previous workshops and as part of the mirror data. These questions had no chronological order or phases. As the discussion in the previous workshop had been on benefits, the checklist started the same way. The questions were also formulated so as to make potential users reflect on what they might have missed or whom they might have forgotten to include, so that there would not be too many questions, and so that they would be able to guide users more implicitly.

The second stimulus inspired a number of reactions, and in the discussion, the participants expressed what they believed was critical and did not work in the checklist as presented to them, and what changes should be made in order to make it work. The participants first reacted to the researchers’ checklist, and then guided the researchers to take notes on a computer on how to amend it.

#### Wrong Start (or What’s the Order?)

The first reaction to the checklist was that the beginning was wrong. The participants seemed to agree that it should not start out with the benefits, but rather with identifying the relevant actors and competences (such as legal experts) both inside and outside the organization who should be part of the process. Understanding the problem or need was also considered to be an important starting point.

“*From my perspective it becomes impossible to answer the first question “Are there well-defined benefits for the organization?” if I have not understood what parts of the organization are affected*” (Julia, case officer).

“*What are the well-defined benefits for the organization? To me this is going about it the wrong way, because it will automatically make me think about my own part in this instead of first identifying the internal and external actors*” (Julia, case officer).

“*When we did this [BRM], we did not work like that. Now we’re using these 30 minutes to identify what stakeholders there are in the upcoming analysis. You don’t know from the start, but will need to find out*” (Sara, IT Unit and BRM project manager).

Or it should start by understanding the problem.

“*I would try to understand the reason and the problem. I found that to be missing* [from the checklist] (Sara, IT Unit and BRM project manager).

“*But I do of course understand that a checklist might never be totally linear, never. You might need to take it step by step and at times go back to prior steps. I understand that. But my first reaction here is that the order is not very logical*” (Julia, case officer).

#### Do Not Decide on the Target Group Too Soon

Another element the participants agreed upon in the discussion was the need not to decide who the target group was and close it too soon. The tendency to tailor specific solutions to a specific target group may lead to wrong decisions.

Julia (case officer): *If we think about this “remote monitoring at night for older people,” we failed. Why only for older people?*
Sara (IT and digitalization unit): *And why only at night?*
Julia (case officer): *Exactly. We failed as early as at that stage with this specific implementation*.
Joan (RAT): *But then you have remote monitoring, taking away everything that will point to a certain group or time or something like that. Because this is more than just giving the night personnel a better deal.*
Julia: *Or the older people*.
Joan: *Or the older people. Yes, but in this case to feel more secure. But it is also about children or people with autism or whatever*.

#### It Is Too Specific and Not Useable: The Need to Be More General

Another element they reacted to was that that checklist was too complex, and was unusable.

“*For me, I always get caught up in details and that makes it too specific. I mean, the fact that the actors are identified by name. (.) the list I see might become unsustainable*… *I’m thinking that the checklist might be difficult to use if you have a lot of boxes that are not used at all, visually confusing* (…) *It should not become a 30-page novel!”* (Julia, case officer).

Keeping a certain level of abstraction was also desirable as it meant it could be adapted to different contexts and their specific categories, as the following two quotes indicate:

“*Even if it [the checklist] will in part be specific for the municipality of [name of the municipality], the idea is that it should be adaptable and generalizable for other municipalities as well*” (Peter, DISK).

“*It cannot be at that level then, because the municipality of [name of the municipality] consists of all administrations and companies, everything. So you will need to find these general categories for the organization, internally and externally, other actors, volunteers. I am thinking civil society. Because they might also be very influential”* (Julia, case officer).

#### Connections Between Benefits Realization Management and the Checklist: Replacing the Project Manager

The discussion then moved on the relationship between BRM and the checklist, and to the fact that they should be complementary, and not overlap. The checklist could help prevent errors or risks associated with the planning process (BRM) or a reminder of something to be done while planning.

“*What do we need to be reminded of in BRM or what can go wrong*? […] T*he function a checklist might have here is if there is no project manager appointed, someone asking questions*… *I mean, instead of a person, is there something asking questions like “Have you done this and this,” so to speak.*” (Klara, researcher).

The BRM project leader, Sara, mentioned that at the beginning of the planning process [BRM] it is important to gather different perspectives and not to work in small groups, but also that at present she is the only one gathering these perspectives. She wanted a process that was more independent from her as project leader. Spontaneously, she raised the idea that the checklist might even replace her:

“*If I’m allowed to speak freely, I want to be*… *I want it to be more people describing this initiative, the need, to gather what comes from the civil society, from the ground level*—*describing it early on in a structured manner (.) I was thinking I could be replaced* [laughter]” (Sara, BRM project leader).

Other participants agreed with this and reinforced the thought.

*“What you are compiling there [in BRM], could be compiled by the group or the people who came up with the initiative”* (Joan, RAT).

This discussion about the researchers’ checklist allowed an improved appropriation of the process. The participants identified problematic elements of the proposed checklist and identified alternatives, this time connected to their own experience and work practices. It was even thought that the checklist might replacing the project leader herself. There was also an attempt to try to make the checklist more usable.

### A New Checklist as a Working Method

At a certain point, the researchers decided to let the participants talk and work alone, and began working on a new paper version of the checklist (see Figure 4 and its translation in Table 2).

**FIGURE 4:** Participants’ paper checklist.

**TABLE 2:** Researchers’ translation of participants’ checklist into a table, organized into different categories.

Steps	Actions	Specifications
**An idea appears**		
**Step 1—Preparation**	Describe the need	
	Describe who needs to be involved	Boundary crossing Co-creation Service design Civil society
	Describe the problem/need/solution to what	
	Target group at the moment	
	Have you found anyone else that has a solution for it at the moment	
**Decision**—**possibly “committee of politicians decision”**—**coordination and prioritization**		
**Step 2—Someone pointed out for leading the initiative**—**project manager or developer (?)**	Update of the stakeholders list	In the organization Also civil society
	Root cause analysis	
	Describe the current workflow	Current system Legal requirements
	Describe the desired workflow and how it affects other actors/organizations, for instance relatives	
	Identify the future target groups	IT system technicians Staff in the unit (förvaltning) Internal ?? use the service?? receiver of the service
	Do a first benefit analysis, “effektmål”	Time to do other things Environment
**Decision**		
**Step 3**—**Same person as above**	Information security classification	
	Check and inform legal officers	
	Material about ?? for bid and “anrop” (when you already have a supplier with a bid) —security perspective	
	Information to ?? IT-architect	
	Information to bid and anrop people	
	Start drafting communication plan	
**Decision**		
**Step 4**—**Decision**—**same person as above**	Update the stakeholder list	
	Get the funding, for the investment and for operating the new solution	See the questions in the checklist produced by the researcher
	Create the solution, including checking what is already on the market	
**Decision**		
**Step 5—Implementation**	Produce a prototype/field trial	Make sure it is user-friendly
**Decision**		
**Step 6**—**Follow-up**		

The participants came up with a six-step process that identified actions to be taken at various stages of the project from the beginning of the project concept to the follow-up. For each step, there could be specifications or principles to follow (these were the researchers’ categorizations, not the participants’). Each phase ended up with a point at which a decision had to be made as to whether to persist with the idea or drop it. It was also decided that the list should have a chronological order.

The agreed process begins with an idea (a solution, a need, a problem, a political agenda, etc.).

In the first stage, which they call “preparation,” someone within or outside the municipal administration advances an idea. During this phase, there is an initial identification of a need or problem, a first definition of the target group and a working group. At this stage, there may more than one target group and more than one solution. Attention is also paid to checking whether anyone within or outside the organization may already have a solution. The involvement of citizens and civil society is important at this stage.

In the second step, the focus moves to a description of current work practices and how future work practices should be. This is also considered to be a way of identifying target groups and checking the stakeholders.

*“Should we put “preparation” and then “next step” here? To describe the current workflow and thoughts about how one would like to work, so you have some preparations here and then step two here. So if we put “Step 1” here and then down here we have “Step 2.” “Describe the current workflow,” or how should I put it? And then “describe desired workflow” or “desired flow” or do you know this already at the “idea” stage?* […] “*Describe the current routine” maybe, or “describe the current workflow,” because then you will find the target groups and if there are more stakeholders*” (Sara, IT Unit and BRM project leader).

In the third step, the initial idea must be fleshed out: other people need to be involved in order to add details to the process (the security coordinator and legal officer, personnel responsible of the bids and for communication need to be involved) and the effects must be specified:

*“What effect will we have? Yes, we might have less transport or we reduce stress because we do not need to*…” (Sara, IT unit and BRM project leader).

The fourth step focuses on creating a solution, finding funds and updating the stakeholders again. In this phase there is an explicit reminder of the questions in the researchers’ checklist. The fifth phase (implementation) and the sixth (follow-up) were mentioned but not developed. The checklist therefore mainly focuses on initiating the process and the successive phases until the solution has been developed.

What was designed was a process in different stages in which there is a progressive definition of the idea with its actors and a progressive formalization and concretization of the process until implementation and follow-up.

One might say that in this process, the checklist partly reproduces the BRM linear dynamic, which consists in having an initial descriptive part (of the problem, of the actors, of the “workflow”), followed by a design/implementation part. The checklist thus emerges in relation to BRM. At the same time, during the discussion the participants mobilized the questions proposed by the researchers in the previous checklist so as to ensure that no important elements had been forgotten, and in particular to update any stakeholders who might be involved. The checklist thus also emerges in relation to the proposed stimulus. A clear connection to these questions was made in step 4 of their checklist, and also during their discussions.

For example, in order to develop step 1, they referred to the researchers’ draft so that they would be certain not to forget anything:

“*Before decisions to proceed, good to check priorities and possibility of coordinating with other initiatives*” (from the researchers’ checklist).

Once again, the discussion on this step 3 was based on the questions presented in the previous checklist around the safety of the technology and its user-friendliness. They seemed to reuse several of our questions, but formulated them differently, as shown in the following quotes:

“*How safe does the technology need to be? It’s about this information safety classification and basic data from the information classification for procurement and ordering. It’s this one*… *the “safety perspective.” So it’s included. And we have another one: “Is the technology user-friendly?” That must be about designing prototypes and*…” (Julia, case officer).

“*There is a question here “Is it necessary to further specify the responsibility of various organizations or professions?” And we added that to it, just from another point of view, to look at more stakeholders*” (Joan, RAT).

It might be said, therefore, that the final checklist is the product of an alignment of different objects: not only the BRM and the researchers’ versions, but also the formal material presented during the workshop. In particular, the checklist developed by the participants maintains the linear approach of the planning tool, while at the same time seeking to add—and also reformulate—certain qualitative dimensions (“how” questions) that emerged from the researchers’ proposals: some “how” questions and in particular the need to update the stakeholders and people to be “listened to” at each stage and the potential target groups.

### The Last Workshop and the Final Digital Checklist

This story was brought to an unexpectedly early end by the COVID outbreak, which made it necessary to call a halt to the physical workshops after the third meeting. In the meantime, the researchers and DISK met Sara (the IT Unit and BRM project leader) on several occasions in order to gain a better understanding of what the BRM model does when organizing new initiatives, and decided to work on the input from the third workshop to develop a digital platform of the checklist, with the help of an information design professional (a former student at the university). Further discussions were therefore held in this group not only to formulate questions in ways that met the practitioners’ needs as expressed in the previous workshops, but also to incorporate the researchers’ insights to be included in the emerging web application, which has spatial limitations. The questions also needed to be as brief as possible in order to enhance their clarity. Considerable energy was also dedicated to determining how to present questions and what visual metaphors to use in order to materialize the idea that the checklist supported a transformational process, rather than an implementation, that might require iteration, and which questions are related to each other at each stage, rather than in chronological order. The final checklist is therefore the result of a re-materialization of the participants’ checklist, to which the researchers and DISK have added their knowledge of the problems entailed by viewing the introduction of technology as a linear process (see Figure 5).

**FIGURE 5:** The final digital version of the checklist.

## Discussion

The aim of this study was to initiate a process of transformational change in a context in which multiple and interdependent practices at the boundaries of different institutions are engaged in performing care for older people, and where WT are used. The research project provided a framework for bringing together practitioners within and outside a municipality in Sweden, as well as older people, in order to develop a new tool for introducing WT. While investments are being made in WT in terms of public discourse and political strategies, the need for new working methods is a central challenge. In order to initiate the transformational process, the study drew its inspiration from the methodology of the CL (Engeström, 1987), which had its origins in Historical and Cultural Activity Theory (CHAT), and which focuses on change and learning as ongoing practical achievements. Building on more recent conceptualizations of practice, and in particular on the idea of work as a sociomaterial accomplishment, we have articulated a method by which change—and its content and forms—is not pre-established, but is produced in the course of the process itself without distinguishing between the subject and object of an activity, but by considering them as co-constituting each other.

The researchers proposed a series of workshops in which initial mirror data were provided to initiate a discussion on the problems and contradictions experienced by participants associated with the introduction of the night camera system. A second stimulus was then proposed by the researchers to initiate a discussion on a possible solution.

The first stimulus—the material collected by the researchers—enabled extensive brainstorming on existing bottlenecks and contradictions in the adoption of WT.

In the first stimulus, the practitioners and older people came together and reacted to the mirror data prepared by the researchers. A number of problematic issues emerged from this first discussion, especially the need to move the focus away from devices and toward new working methods and practices. In particular, attention was drawn to a lack of coordination among the different units of the administration and outside the organization, specifically the involvement of external experts (RAT and DISK) and end users (older people). The checklist was initially identified as a potential solution. This tool is based on a simple principle, which is “not to forget,” and is commonly used in a wide variety of sectors—from industries in the engineering sector to public services—to help coordination of highly complex work activities.

In this phase, the process was led mainly by the researchers and the data and material they had gathered and organized for the purpose.

The process continued with an exploration of different aspects that should be integrated into the solution, such as how to collect and deal with and prioritize initiatives and ideas in the area of WT, what principles should inspire the process of adopting WT, and last but not least what kind of profile would be the most suitable to lead the process. Doubts emerged about whether managers are the most suitable candidates for this role.

The checklist thus took the form of a solution through successive materializations and encounters with other objects that emerged during the process itself.

In the second stimulus, the checklist proposed by the researchers was challenged by the participants on a different basis—because it did not provide relevant questions, because it was not in a particular order, because it was not sustainable—and they decided to develop their own (albeit one connected to the researchers’ version). As Engeström claims, resisting interventionists’ proposals and proposing something new represents an important turning-point in a sociomaterial configuration and in the distribution of power among actors. He writes: “The participants take actions that redefine and transform the initially planned object of the learning effort, thus changing the entire course of the process and forcing the interventionists to redefine their script. The deviations and negotiations are important instances of emerging transformative agency among the participants (Engeström and Sannino, 2012 in Engeström et al., 2014: 123).” The decision not to continue working on the researchers’ checklist marked a deviation by the participants from the interventionists’ process design or script (Engeström et al., 2014).

In this phase, BRM—a systematic planning tool that was already in use at the municipality—came on the scene as a new actor, and was welcomed by the participants as a pragmatic, “smart” tool. In this way, a new alignment of actors was produced whereby the checklist—the main solution—and BRM began to be thought about together. The new structural materialization of the checklist produced by the participants was similar to that of BRM. This clearly produced a new sociomaterial alignment in which the checklist emerged as complementing or integrating the planning tool, which proposed a somewhat linear and idealized approach to management planning (Breese, 2011) and did not encourage the involvement of external actors to the same extent. This is not all, however: there was even the idea that the checklist should take a leading role in the process of adopting WT, substituting the manager and his/her power to control the process in favor of a more collective way of appropriating and leading it. In this phase the researchers felt that the process was moving toward a dynamic of traditional and rationalistic planning process, but they let the process be and followed the actors.

In the final part of the process, the new materialization of the checklist—the digital version—was produced whereby in the end two different logics were combined in the final tool. There was a need to control and rationalize a planning process on the one hand, and the need to amend it in order to move closer to actual working practices within the administration and to keep the connections of a complex and composite work when initiating WT on the other. The checklist is the result of a specific alignment of actors during the process and their interactions. It has been conceived as a dialectical process between the researchers’ way of framing the situation and problem and the practitioners’ method, with their own practices and sense-making. In the first workshop, the researchers retained power and control because it was they who presented tangible texts and wrote new ones. Later, “handing the pen over” to the practitioners when they were asked to react to the original checklist and produce their own after the second stimulus also meant losing control and their priority position when it came to formulating solutions. Each time something written was produced it gave rise to reactions and resistance, as it did not completely meet the others’ expectations. When the researchers proposed their checklist, the practitioners disagreed, even though they incorporated some of the original text in their reformulation. On the other hand, when the practitioners presented their text, the researchers and DISK reacted, because they viewed the practitioners as being caught up in discourses of linearity and solutions, rather than being open to problematizing and constructing something different based on these issues.

The final product represents a path between the different ways of constituting and articulating practices, and has a completely different form from what is customarily used in organizations, which may make it easier to see its value. It also materializes the need for a variety of actors, within or outside an organization, to participate in the introduction of WT, and thus reminds a user and enables her/him to invite different actors into the process where required. When in use, the checklist may therefore create the premise for assembling actors in the process of introducing WT, and may help keep them connected throughout the process.

## Conclusion: On Organizational Change and Welfare Technologies

This study has described a transformative process that leads to the development of a solution—a checklist—to support cooperative work in the context of working with change when introducing new technologies. The new device/solution is the result of a process in which practitioners, researchers and contextual objects interacted and became one. The process from which the checklist emerged was in the form of successive back-and-forth movements among different objects that the practitioners and researchers interacted on.

The methodology of intervention research that was proposed is not strictly speaking a way of “studying groups” (as this special issue called for); rather, it is a means of initiating a co-creation process at the crossroads of different communities of people—practitioners, older people and researchers—and materialities (Orlikowski, 2009). In the methodology that was adopted—which was inspired by the CL (Engeström, 1987)—the solution was not pre-defined and the transformational process was not traced beforehand. The researchers and practitioners engaged in an iterative process the result of which was not known in advance, as will the actors—human and non-human—who will participate in it and the role they will play.

The checklist and the contradictions that emerged from it represent a way of moving the focus of attention away from a multiplicity of problems and principles to the development of more suitable concrete propositions that tie in with practitioners’ work experience and practice. However, while the checklist appeared from the outset to be a potential tool on which actors could work, the planning tool (BRM) emerged as an actor in the process. This led to a reorientation of discussions on the checklist in relation to this powerful pre-existing rationalistic framework (Breese, 2011). In this process, the zone of proximal learning (Engeström, 2000) resides in the interstices of this rational and linear framework—which is provided by the planning tool, and more generally by the administrative organizational infrastructure—which it is hard for practitioners to make visible and for participants to question.

The process also speaks of agency formation, in the sense that the practitioners in the process are the same people who pick up a pencil and re-design their own tool and working method, using their own practices, motives and sense-making as a starting point. To what extent this leads to a complete reconceptualization of the object of the activity, as the CL aims to, is something this study cannot determine as COVID—another emerging actor in this research process!—made it impossible to follow the application of the checklist to concrete welfare technology initiatives (which could be the subject of another study).

In any case, as Engeström claims (Virkkunen and Newnham, 2013), the focus of attention in transformative processes does not reside in the solution itself—the final checklist in this case—but in the dialectical work to overcome its contradictions and through its different materializations and re-materializations that leads to its development. It is in this sense that the methodology that has been adopted in this study raises interesting questions for further research in the area of organizational change, where several stakeholders and professions are involved in general, and more specifically in relation to WT. In this regard, Engeström (2007) has returned to the idea of community [and in particular the idea of “community of practice” (Lave and Wenger, 1991)] to point out that in contemporary society, there is a need to study work and collaboration within communities that are more dispersed and loose, but also highly interdependent, as is the case here.

The transformative process we have suggested makes it possible not to work on general solutions, but to let practitioners—with the support of researchers—generate their own solutions, starting out from their specific and composite organizational practices, networks, ambiguities, uncertainties and tacit knowledge connected to care work. This is the sense in which change is proposed as a specific and contextual *agencement* (Gherardi, 2019) of human and material actors. In this process, we see a reconfiguration of the sociomaterial alignment of actors that leads to a new understanding and knowledge of the solution that is outlined. In this reconfiguration, we also see different displacements of power relations: from the researchers to the practitioners who reinvent the initial checklist, to BRM and then to the checklist, whose agency is meant to replace the manager’s role.

The iterative process we have shown suggests that WT are a matter of local and multiple *agencements* of humans and materials. This proposed change in the adoption of WT implies negotiation among sociomaterial practices at the organizational boundaries whereby power and agency are temporal stabilizations, and are always distributed between the social and the material.

## Data Availability Statement

The original contributions presented in the study are included in the article/supplementary material, further inquiries can be directed to the corresponding author/s.

## Ethics Statement

Ethical review and approval was not required for the study on human participants in accordance with the local legislation and institutional requirements. Written informed consent for participation was not required for this study in accordance with the National Legislation and the Institutional Requirements.

## Author Contributions

All authors listed have made a substantial, direct, and intellectual contribution to the work, and approved it for publication.

## Conflict of Interest

The authors declare that the research was conducted in the absence of any commercial or financial relationships that could be construed as a potential conflict of interest.

## Publisher’s Note

All claims expressed in this article are solely those of the authors and do not necessarily represent those of their affiliated organizations, or those of the publisher, the editors and the reviewers. Any product that may be evaluated in this article, or claim that may be made by its manufacturer, is not guaranteed or endorsed by the publisher.

## Footnotes

1
https://nordicwelfare.org/en/welfare-policy/welfare-technology

2
https://nordicwelfare.org/en/publikationer/welfare-technology-tool-box/

3 Some of these interviews and observations were conducted in the framework of the IVRIS sister project Sins-Developing the capacity of leading technology-related social innovation in cooperation (Vinnova, 2017–2019).

4 Incidentally, in IVRIS’ sister project SINS, the idea of a checklist had already been raised by a project management team from the same municipality working on the adoption of welfare technology.

5 See a description here of this model inspired by design thinking https://www.designcouncil.org.uk/news-opinion/double-diamond-universally-accepted-depiction-design-process.

6
http://wiki.doing-projects.org/index.php/Double_Diamond_in_Project_Management
